This article has been retracted.

# The hematological impact of umbilical cord milking versus delayed cord clamping in premature neonates: a randomized controlled trial

**DOI:** 10.1186/s12884-022-05046-7

**Published:** 2022-09-19

**Authors:** Hytham Atia, Ahmed Badawie, Osama Elsaid, Mahmoud Kashef, Nourhan Alhaddad, Mohamed Gomaa

**Affiliations:** 1 Faculty of Medicine, Zagazig University, Zagazig, Sharkia Egypt; 2 Armed Forces Hospitals Southern Region, King Faisal Military City Hospital, Base-villa 68, King Faisal military city, 62417-8183 Khamis Mushait, Kingdom of Saudi Arabia; 3 Faculty of Medicine, October 6 University, Cairo, Egypt; 4 Al Ahmady Hospital, Madina, Kingdom of Saudi Arabia

**Keywords:** Cord milking, Deferred clamping, Hematocrit, Preterm, Placental transfusion

## Abstract

**Background:**

The hematological impact of umbilical cord milking (UCM) was compared to that of delayed cord clamping (DCC) as a faster placental transfusion technique for preterm neonates (between 24 and 34 + 6 weeks gestation). A comparison of important neonatal morbidities was also made.

**Methods:**

This was an open-label randomized trial conducted from June 8, 2017, to April 22, 2019. Two hundred patients with preterm deliveries (24 and 34 + 6 weeks gestation) were assigned to the DCC or UCM group at random at a ratio of 1:1. The study power was 80% for a difference in the hematocrit value of 3% and Hb value of one gram, and an alpha error of 0.05.

**Results:**

The following variables were analyzed in the comparison of UCM vs. DCC: first draw hemoglobin: 17.0 ± 1.9 vs. 16.8 ± 1.8 gm/dl (95% CI -0.75–0.29, P 0.383); first draw hematocrit: 55.6 ± 6.4 vs. 55.2 ± 6.4% (95% CI -2.18–1.38, P 0.659); peak hematocrit: 56.9 ± 6.4 vs. 56.3 ± 6.7% (95% CI -2.41–1.26, P 0.537); the need for respiratory assistance (47% vs. 30%, P 0.020), inotropes (16% vs. 6%, P 0.040), and blood transfusion (26% vs. 12%, P 0.018); and the occurrence of intraventricular hemorrhage (9% vs. 5%, P 0.407), necrotizing enterocolitis (6% vs. 2%, P 0.279), sepsis (25% vs. 15%, P 0.111), and neonatal death (13% vs. 4%, P 0.40).

**Conclusion:**

UCM facilitated a rapid transfer of placental blood equivalent to that of DCC for premature neonates. However, it resulted in increased rates of interventions and morbidities, especially in extremely preterm neonates.

**Trial registration:**

The clinical trial was registered on May 10, 2017, with registration number (NCT03147846).

## Tweetable abstract

Cord milking allowed rapid transfer of comparable blood amounts, but with increased interventions and morbidities.

## Introduction

Placental transfusion enhancement secures an additional 10 to 30 mL/kg of blood and approximately 20 to 30 mg/kg of iron for preterm neonates [1]. This volume supports the physiological fetal to neonatal circulatory transition process compared to immediate cord clamping, which deprives newborns of an important volume of blood to endure the major changes in pulmonary and umbilical circulations, especially in preterm neonates [2]. Different methods enhancing placental transfusion were used, including deferred umbilical cord clamping (DCC) and successive umbilical cord milking (UCM) or stripping [3].

The beneficial impacts of DCC compared to immediate cord clamping occur through increasing the circulatory blood volume. This leads to better blood pressure, a reduced need for inotropes, a reduced need for transfusion, and a reduced incidence of necrotizing enterocolitis (NEC), intraventricular hemorrhage (IVH), and early death before discharge [4–7]. DCC is an intervention recommended by the Royal College of Obstetricians and Gynecologists for both full-term and premature neonates [3]. Similarly, the American College of Obstetricians and Gynecologists recommends DCC for all preterm newborns [8].

The time required to accomplish DCC might expose susceptible preterm neonates to delayed resuscitation and hypothermia. This important time-lapse could be minimized if UCM was used instead, before respiratory support, especially for apneic preterm infants [9]. Fogarty et al. [10] highlighted the need for further clinical trials to investigate the beneficial impact of UCM versus DCC in premature neonates.

The study's main goal was to assess the impact of UCM compared to DCC on the hematological index in preterm newborns. Secondary variables of interest were included to assess the composite morbidities between both methods and the safety of UCM as a feasible alternative to DCC.

## Patients and methods

### Study setting

This was an open-label randomized controlled trial primarily comparing the hematological impacts of UCM and DCC for preterm neonates born at 24^+0^ weeks to 34^+6^ weeks gestation. Institutional Review Board approval was obtained from the research ethics committee of the Armed Forces Hospital Southern Region, KSA (Registration Number: H-06-KM-001). The trial was registered at clinicaltrials.gov with registration number {NCT03147846 (10/05/2017)}, and the CONSORT guidelines [11] were followed. All included mothers were counseled about the predicted placental transfusion benefits and the process of the study using both transfusion methods. After agreeing to participate, they prospectively signed informed consent forms.

The study setting was in the Armed Forces Hospitals Southern Region, KSA; the attending obstetricians recruited patients from June 8, 2017, through April 22, 2019, and were responsible for obtaining informed consent. Recruitment stopped once the targeted sample size was achieved.

The inclusion criteria were individuals with a singleton pregnancy who were admitted with preterm labor between 24^+0^ weeks and 34^+6^ weeks gestation. The exclusion criteria were as follows: multifetal pregnancy, diagnosed congenital anomalies, fetal anemia, considerable antepartum hemorrhage, and category III cardiotocography tracing (Fig. 1).

**Fig. 1:** Study flow chart

The simple random sequence was produced using the random sequence generator method on the website https://www.random.org/sequences, with a one-to-one allocation ratio into two separate columns for either group. The first group was subjected to the DCC protocol, in which umbilical cord clamping was deferred for 45–60 s while the baby was at/below the level of the placenta (over the side of the operating table during cesarean delivery or below the maternal pelvis during vaginal delivery). The second group was subjected to the UCM protocol; the cord was left intact, and then 4–5 strips were placed with the thumb and forefinger from the proximal (maternal) end of the cord (as proximal as possible) toward the baby's abdomen. The stripped segment was approximately 20 cm, with a speed of 20 cm over 2 s and 2 s between each stripping, keeping the baby at the level of the placenta. These maneuvers were adapted from earlier similar studies [12, 13]. The allocation sequence cards, including the random number sequence and the requested intervention, were masked using sealed separate envelopes. The selected envelope was opened by the obstetric team just before the procedure. After intervention, the mother/infant ID was on the same card and collected for follow-up, and the selected intervention was also stated in the delivery notes. After the start of the trial, no important changes were made in the methodology.

Principal investigators collected and processed all relevant maternal data, delivery data, neonatal outcome data, and composite morbidity data through an electronic database.

### Sample size calculation

The sample size was calculated using G*Power 3.1.9.2 software and an online sample size calculator (https://clincalc.com/stats/samplesize.aspx). An a priori power analysis for a two-tailed study comparing independent means was performed, with an alpha error of 0.05, a power of 80%, a one-to-one allocation ratio to detect a 3% difference ± 7.5% standard deviation (SD) in the hematocrit value or a difference in the Hb value of one gram ± 2.5 g SD between both study groups as primary hematological outcomes. The least required sample size for both parameters was 196 subjects, and the authors decided to collect 200 participants for the study. The proposed difference in primary outcomes used in the calculation was indirectly determined through the estimated differences in the hematocrit value between both the DCC and UCM groups in comparison to immediate cord clamping, as stated in earlier studies [13–15].

### Statistical methods

Statistical analysis was performed using IBM SPSS version 25 [IBM© Corp., Armonk, NY]. Kolmogorov‒Smirnov and Shapiro‒Wilk tests were used to test the normality of the distribution of the numerical data. Normally distributed data are presented as the mean ± standard deviation (SD), and between-group differences were calculated using independent samples t tests. Skewed data are presented as the median and interquartile range (IQR) and between-group differences were calculated nonparametrically using the Mann‒Whitney U test. Categorical data are presented as numbers and percentages (%), and between-group differences were calculated using the chi-squared test or Fisher's exact test as appropriate.

For comparison of composite morbidity, the collected study population was stratified into 3 subgroups according to gestational age at delivery: 24^+0^–27^+6^ weeks, 28^+0^–31^+6^ weeks, and 32^+0^–34^+6^ weeks. Due to the clear mismatch in neonatal numbers of the three age groups, we performed Chi square post hoc testing after Bonferroni adjustment [16].

Binary regression analysis was performed to test the gestational age at delivery, delivery mode, and method of transfusion as independent predictors of the major morbidities, including severe IVH, NEC, and retinopathy. None of them proved to be significant predictors. Similarly, patients were divided based on delivery mode, and outcomes were matched between the DCC and UCM groups without significant differences (Tables are not included).

## Results

The maternal demographic data were comparable in both groups regarding age, parity, level of antenatal care, distribution of associated medical disorders, and incidence of preterm premature rupture of membranes (Table 1).

**Table 1:** Maternal demographic and delivery outcome data

	**Total** **(*n* = 200)**	**Deferred cord clamping (*n* = 100)**	**Cord milking** **(*n* = 100)**	*P***- value**
Maternal age (years)	29.8 ± 6.9	28.8 ± 6.6	30.8 ± 7.1	0.045^*^
BMI (kg/m^2^)	30.2 ± 5.6	28.9 ± 4.4	31.5 ± 6.3	0.001^*^
Parity	2 (0–4)	0 (0–3)	2 (0–4)	0.106
Level of antenatal care				
Unbooked	50 (25%)	26 (26%)	24 (24%)	0.529
Less than 4 visits	68 (34%)	37 (37%)	31(31%)	
4–8 visits	82 (41%)	37 (37%)	45 (45%)	
Medical disorders	15 (7.5%)	7 (7%)	8 (8%)	0.435
Diabetes mellitus	7 (3.5%)	4 (4%)	3 (3%)	
Hypertensive disorders	6 (3%)	2 (2%)	4 (4%)	
Sickle cell disease	2 (1%)	1 (1%)	1 (1%)	
Preterm premature rupture of membranes	59 (29.5%)	36 (36%)	23 (23%)	0.062
Gestational age (weeks)	31.9 ± 2.4	32.1 ± 2.2	31.4 ± 2.5	0.022*
24- < 28	15 (7.5%)	5 (5%)	10 (10%)	0.037*
28- < 32	52 (26.0%)	20 (20%)	32 (32%)	
32-< 35	133 (66.5%)	75 (75%)	58 (58%)	
Birth weight (gram)	1677 ± 519	1781 ± 483	1573 ± 534	0.004*
Arterial blood PH	7.2 ± 0.08	7.2 ± 0.09	7.2 ± 0.08	0.056
PH less than 7.1	3 (1.5%)	3 (3%)	0	0.081
Apgar score				
At 1 min	7 (6–8)	7 (6–8)	7 (5–8)	0.061
At 5 min	8 (7–9)	8 (8–9)	8 (7–9)	0.061
Score ≤ 6 at 1 min	25 (12.5%)	11 (11%)	14 (14%)	0.521
Score ≤ 6 at 5 min	9 (4.5%)	3 (3%)	6 (6%)	0.306
Mode of delivery				
Vaginal	77 (38.5%)	56 (56%)	21 (21%)	0.000*
Cesarean before labor onset	49 (24.5%)	13 (13%)	36 (36%)	
Cesarean after labor onset	74 (37.0%)	31 (31%)	43 (43%)	
Indication for delivery				
Spontaneous	169 (84.5%)	89 (89%)	80 (80%)	0.079
Induced	31(15.5%)	11 (11%)	20 (20%)	
Uterotonics				
Syntocinon only	196 (98%)	99 (99%)	97 (97%)	0.259
Syntocinon + other ecbolic	4 (2%)	1 (1%)	3 (3%)	
Blood loss				
After vaginal delivery	211 ± 100	206 ± 98	226 ± 109	0.448
After cesarean	535 ± 142	506 ± 67	542 ± 212	0.053
Postpartum hemorrhage	4 (2%)	0	4 (4%)	0.121
Time till cord clamping (seconds)	43.4 ± 19.6	62.8 ± 1.6	24.1 ± 3.5	0.000*
Maternal sepsis	3 (1.5%)	0	3 (3%)	0.316
Antepartum sepsis	0	0	0	
Intrapartum sepsis	1 (0.5%)	0	1 (1%)	
Postpartum sepsis	2 (1%)	0	2 (2%)	

Data are presented as mean ± standard deviation, number (percentage) and median (interquartile range) as appropriate

*n* Number, *BMI* Body mass index

^*^ Statistically significant

Deliveries with lower gestational age groups were significantly more prevalent in the UCM group than in the DCC group {(10 vs. 5 neonates between 24^+0^- 27^+6^ weeks gestation) & (32 vs. 20 neonates between 28^+0^- 31^+6^ weeks gestation), respectively}. In the UCM group, this led to a significantly lower birth weight (1573 ± 534 g vs. 1781 ± 483 g, respectively), significantly higher need for assisted breathing (47% vs. 30%, respectively), and slightly longer hospital stay (29.3 ± 28.6 vs. 21.8 ± 24.9 days, respectively). In addition, this might have led to a significantly higher frequency of cesarean sections (CSs) for the same group {(36% vs. 13% with CS before labor onset) & (43% vs. 31% with CS after labor onset)} (Tables 1 and 2).

**Table 2:** Neonatal outcome

	**Total (*n* = 200)**	**Deferred cord clamping (*n* = 100)**	**Cord milking (*n* = 100)**	***p*- value**
Neonatal gender				
Male	123 (61.5%	60 (60%)	63 (63%)	0.663
Female	77 (38.5%)	40 (40%)	37 (37%)	
First draw Hemoglobin (gm/dl)	16.9 ± 1.9	16.8 ± 1.8	17.0 ± 1.9	0.383
First draw hematocrit value (%)	55.4 ± 6.4	55.2 ± 6.3	55.6 ± 6.4	0.659
Polycythemia	20 (10%)	10 (10%)	10 (10%)	1.000
Peak hematocrit value (%)	56.6 ± 6.6	56.3 ± 6.7	56.9 ± 6.4	0.537
Day 1 bilirubin (gm/dl)	4.6 ± 2.1	4.8 ± 2.2	4.4 ± 2.1	0.198
Peak bilirubin (gm/dl)	7.9 ± 3.4	8.1 ± 3.1	7.8 ± 3.6	0.541
First breath				
Spontaneous	123 (61.5%)	70 (70%)	53 (53%)	0.020^*^
Assisted	77 (38.5%)	30 (30%)	47 (47%)	
First breath				
Before cord clamping	155 (77.5%)	100 (100%)	55 (55%)	0.000^*^
After cord clamping	45 (22.5%)	0	45 (45%)	
Need for tactile stimulation	109 (54.5%)	48 (48%)	61 (61%)	0.065
Oropharyngeal suction	99 (49.5%)	43 (43%)	56 (56%)	0.066
Bag and mask ventilation	81 (40.5%)	34 (34%)	47 (47%)	0.061
CPAP	110 (55%)	49 (49%)	61 (61%)	0.088
Intubation	46 (23%)	17 (17%)	29 (29%)	0.044^*^
Mechanical ventilation	67 (33.5%)	27 (27%)	40 (40%)	0.051
Temperature	36.8 ± 0.2	36.8 ± 0.2	36.8 ± 0.3	0.181
< 36.5 C˚	8 (4%)	3 (3%)	5 (5%)	0.721
> 36.5- 37.5 C˚	192 (96%)	97 (97%)	95 (95%)	
Surfactant	61 (30.5%)	24 (24%)	37 (37%)	0.046^*^
Duration till hospital discharge	25.5 ± 27.1	21.8 ± 24.9	29.3 ± 28.6	0.049^*^

Data are presented as mean ± standard deviation, number (percentage) and median (interquartile range) as appropriate

*n* Number, *CPAP* Continuous positive airway pressure

^*^ Statistically significant

There were no significant changes in the postpartum hemorrhage risk, need for ecbolics, blood loss amount (using visual estimation as per pictorial guidelines) [17], or maternal sepsis. The mean time-lapse until cord clamping with UCM (24.1 ± 3.5 s vs. 62.8 ± 1.6 s) and DCC (95% CI 38.0–39.53, P 0.000) halved the duration until starting neonatal resuscitation (Table 1).

Similar to DCC, UCM enhanced the transfusion volume; this appeared through comparable results of the first draw hemoglobin concentration {17.0 ± 1.9 vs. 16.8 ± 1.8 gm/dl, respectively (95% CI -0.75–0.29, P 0.383)} and the first draw hematocrit value {55.6 ± 6.4% vs. 55.2 ± 6.4%, respectively (95% CI -2.18–1.38, P 0.659)}. The same findings were found for admission temperature {36.8 ± 0.3 vs. 36.8 ± 0.2 °C, respectively (95% CI -0.02–0.11, P 0.181)}. Later, both groups were comparable regarding peak hematocrit values {56.9 ± 6.4% vs. 56.3 ± 6.7%, respectively (95% CI -2.41–1.26, P 0.537)} and peak bilirubin levels {7.8 ± 3.6 gm/dl vs. 8.1 ± 3.1 gm/dl, respectively (95% CI -0.65–1.33, P 0.541)} (Table 2).

The UCM arm, compared to the DCC arm, seemed to be exposed to increased intervention rates, including the need for breathing assistance (47% vs. 30%, P 0.020), surfactant (37% vs. 24%, P 0.065), inotropes (16% vs. 6%, P 0.040) and blood transfusion (26% vs. 12%, P 0.018) (Table 2). This in part is due to the lower gestational age in the UCM arm (42 vs. 25 neonates below 32 weeks gestation). Nevertheless, the role of UCM in such an increase is unclear.

Regarding neonatal complications, intraventricular hemorrhage (IVH) affected 9% of UCM neonates, compared to 5% in the DCC group (P 0.407). Severe forms of IVH (grades III & IV) were more frequent in the UCM group (4% vs. 1%, P 0.369), all occurring in neonates below 32 weeks. The UCM arm showed a similarly higher frequency of other morbidities compared to the DCC arm. This included necrotizing enterocolitis (NEC) (6% vs. 2%, P 0.279), retinopathy of prematurity (6% vs. 4%, P 0.748), late-onset neonatal sepsis (25% vs. 15%, P 0.111), and death before discharge (13% vs. 4%, P 0.40). Such differences, although not statistically significant, should receive attention (Table 3). Unfortunately, the study size was underpowered for neonatal morbidities.

**Table 3:** Neonatal morbidities/ mortality

	**Total (200)**	**24- < 28 weeks (15)**			**28- < 32 weeks (52)**			**32- < 35 weeks (133)**		
		**DCC (5)**	**UCM (10)**	***P*- value**	**DCC (20)**	**UCM (32)**	***P*- value**	**DCC (75)**	**UCM (58)**	***P*- value**
Neonatal jaundice	146 (73%)	2 (40%)	5 (50%)	0.714	15 (75%)	25 (78%)	0.795	53 (71%)	46 (79%)	0.257
Phototherapy	133 (66.5%)	2 (40%)	5 (50%)	0.714	13 (65%)	24 (75%)	0.439	45 (60%)	44 (76%)	0.054
Need for inotropes	22 (11%)	1 (20%)	6 (60%)	0.143	4 (20%)	8 (25%)	0.677	1 (1.3%)	2 (3.4%)	0.415
Need for transfusion	38 (19%)	3 (60%)	7 (70%)	0.699	4 (20%)	11 (34%)	0.266	5 (6.7%)	8 (14%)	0.170
Intraventricular hemorrhage (IVH)	14 (7%)	3 (60%)	2 (20%)	0.121	2 (10%)	6 (19%)	0.395	0	1 (1.7%)	0.254
Severe IVH (grade III, IV)	5 (2.5%)	1 (20%)	1 (10%)	0.591	0	3 (9.4%)	0.158	0	0	NA
Periventricular leukomalacia	3 (1.5%)	0	0	NA	0	1 (3.1%)	0.425	1 (1.3%)	1 (1.7%)	0.854
Necrotizing enterocolitis (NEC)	8 (4%)	1 (20%)	2 (20%)	1.00	1 (5%)	1 (3.1%)	0.732	0	3 (5.2%)	0.046
Late onset Neonatal Sepsis	40 (20%)	3 (60%)	7 (70%)	0.699	10 (50%)	10 (31%)	0.176	2 (2.7%)	8 (14%)	0.016*
Retinopathy	10 (5%)	3 (60%)	3 (30%)	0.264	1 (5%)	3 (9.4%)	0.565	0	0	NA
Patent ductus arteriosus medically managed	33 (16.5%)	3 (60%)	3 (30%)	0.264	4 (20%)	12 (38%)	0.183	7 (9.3%)	4 (6.9%)	0.613
Patent ductus arteriosus need surgical management	1 (0.5%)	0	1 (10%)	0.464	0	0	NA	0	0	NA
Neonatal death before discharge	17 (8.5%)	2 (40%)	5 (50%)	0.714	2 (10%)	6 (18.8%)	0.395	0	2 (3.4%)	0.105

Data are presented as number (percentage)

*n* Number, *DCC* Deferred cord clamping, *UCM* Umbilical cord milking

^*^ Statistically significant

## Discussion

Placental transfusion enhancement became a recommended practice for both full-term and preterm deliveries [3, 8]. Performing the DCC method takes approximately 60 s to allow transfer of the desired placental blood amount to newborn circulation. The time used to perform DCC could delay vital neonatal resuscitation, an important time for premature neonates who require it [9, 18]. This randomized trial showed that UCM could achieve the same goal in a significantly shorter duration with almost the same hematological values. However, worrisome impressions regarding hemodynamic instability in addition to other morbidities after UCM are acknowledged.

In this trial, UCM required a mean duration of 24 s until cord clamping, less than half the duration needed for DCC. This significant reduction allowed for faster neonatal resuscitation by neonatologists.

We adopted hematological value comparisons as surrogate indicators for transfusion volume. UCM showed similar or slightly higher elevation in this indicator compared to DCC. These results are consistent with those of Shirk et al. [19] and Katheria et al. [20]. Five strips of UCM allowed the active transfer of placental blood in a volume comparable to that of passive DCC within a significantly shorter duration.

In their meta-analysis, Backes et al. [21] found a mean weighted difference of -1.14 in the blood transfusion frequency in the DCC group when compared to the immediate clamping group (6 studies, 95% CI -2.01–0.27, *P* < 0.01). Similar findings were addressed by Fogarty et al. [10] (reduction of 10% (95% CI 6 to 13%, *P* < 0.00001)).

The amount of enhanced transfusion was not linked to a critical elevation in peak bilirubin levels or a significant rise in the occurrence of neonatal jaundice or phototherapy in the three gestational age strata for UCM compared to DCC (Table 2). Our findings are supported by those of other researchers reflecting the safety of either method in this aspect [12, 19].

It was notable that neonates in the UCM arm were in need of more resuscitative procedures in the form of respiratory assistance (P 0.020) and surfactant therapy. The higher number (42 vs. 25) of neonates with a gestational age below 32 weeks and the shorter duration given for neonates in the UCM group to take a spontaneous breath before the start of resuscitation compared to that the DCC group might be the reason. However, this higher trend should alert us regarding the compatibility of UCM with the physiological adaptation of extremely premature neonates.

In the UCM arm, 26% of the neonates needed blood transfusion compared to 12% in the DCC arm (P 0.018). This trend was notable along the three gestational age strata (Table 3). In line with the previous findings, the overall increased need for inotropes (16% vs. 6%, P 0.040) should attract attention that UCM might be less physiological than DCC, which seemed more beneficial. This was more evident in the 24^+0^- 27^+6^ weeks stratum, where six neonates (60%) in the UCM arm required inotropes for neonatal hypotension compared to only one (20%) in the DCC arm (P 0.143). The notably fewer number of neonates recruited in such a gestational age category requires caution when implementing the results for neonates below 28 weeks gestation. Despite being statistically insignificant, we can say that UCM was less efficacious than DCC in supporting hemodynamic stability for preterm neonates. The benefits of either method in reducing hemodynamic instability and improving cardiac output, cerebral perfusion, and tissue oxygenation have been highlighted in multiple studies [2, 15, 22]. Knol et al. [18] expressed the contradictions in the physiological perspectives of UCM as an enhanced transfusion method compared to DCC. They proposed the notion of physiological-based cord clamping that allows the incorporation of clamping timing into infant resuscitation to decide the optimal time.

Different studies have addressed the protective value of DCC against IVH and NEC in either term or preterm neonates compared to immediate clamping [10, 14]. The same protective value was addressed by a few studies for UCM with no increased adverse effects on preterm neonates [23, 24]. In this trial, IVH affected 9% of the neonates in the UCM group compared to 5% in the DCC group. Severe IVH (grades III & IV) affected four (4%) of the neonates in the UCM group compared to one (1%) neonate in the DCC group, all below 32 weeks gestation. This suggests that, when compared to DCC, UCM was linked to a higher incidence of IVH. Katheria et al. [20] terminated their trial early because the UCM group had a considerably greater incidence of severe IVH compared to the DCC group in neonates below 32 weeks gestation. They related their findings to the increased fragility and high vascularity of the germinal matrix that increases the susceptibility of hemorrhage with UCM. One of the trial limitations is the low percentage of neonates below 32 weeks gestation {67 neonates (33.5%)}. Our findings are in agreement with the warning findings of Katheria et al. [20] regarding the risk of severe IVH when performing UCM for extremely preterm neonates; further well-designed studies might be required for more clarification.

Neonates who received UCM experienced a similar higher incidence of the following morbidities compared to those who received DCC: NEC (6% vs. 2%), retinopathy of prematurity (6% vs. 4%), late-onset neonatal sepsis (25% vs. 15%), and patent ductus arteriosus (20% vs. 14%). These nonreassuring findings were statistically insignificant, but still increasing worries about the safety of UCM and led to a significantly higher incidence of neonatal death before discharge (13% vs. 4%, P 0.40) (Table 3).

Preterm neonates might need expedited initiation of resuscitation without delay. Although UCM seemed more favorable in this regard, the higher incidence of interventions and major morbidities raises serious concerns regarding its safety as an alternative method to DCC, especially for extremely preterm neonates below 28 weeks gestation.

The main strength of our trial is the randomized controlled trial design with adequate power for the primary outcomes and a complete sample size for preterm neonates. In addition, there was a standardized design regarding the delivery protocol, the use of ecbolics, and the newborn's level in proportion to the maternal level during placental transfusion.

The limitations of this trial include not performing ad hoc stratification based on the gestational age group, which would allow an equal presentation of the three groups. This led to relatively fewer extremely preterm neonates being included (24^+0^- 27^+6^ weeks gestation). Only 15 neonates (7.5%) were included and unequally distributed in both arms of the study. In turn, this might have affected the reliability of our findings for this age group, despite our findings being supported by findings of previous studies for the same category [19, 25]. The stratification of study groups according to gestational age or the restriction of the study for specific age subgroups should be considered during the design of any future trials. Additionally, being underpowered for the detection of less frequent major morbidities (such as IVH, retinopathy, NEC, and neonatal mortality) made the noted difference in the occurrence of such serious complications between both arms of limited value. Nevertheless, our findings are consistent with the safety concerns raised by Katheria et al. [20] and recommend against performing UCM for neonates below 28 weeks gestation. In fact, such morbidities need a much larger sample size that seems nonapplicable for randomization in addition to the ethical aspects. Safety concerns regarding UCM and severe IVH seem to be the most relevant area for further assessment.

## Conclusion

UCM facilitated a rapid transfer of placental blood equivalent to that of DCC. However, it resulted in increased rates of interventions and morbidities, especially in extremely preterm neonates.

## Data Availability

De-identified data is available from the corresponding author on reasonable request.

## Abbreviations

DCC: Deferred cord clamping
UCM: Umbilical cord milking
NEC: Necrotizing enterocolitis
IVH: Intraventricular hemorrhage
CS: Cesarean section
IQR: Interquartile ratio
NICU: Neonatal intensive care unit
BMI: Body mass index
CI: Confidence interval
